# Probe into the Low-Carbon Economic Environment Challenges and Opportunities of Textile and Garment Export

**DOI:** 10.1155/2022/6043903

**Published:** 2022-09-30

**Authors:** Ronghua Chang, Shaoying Zhu

**Affiliations:** College of Business, Shanxi Datong University, Datong, Shanxi 037009, China

## Abstract

Ecological and environmental protection is the main problem of China's economic construction. As one of the high-energy-consuming industries, the traditional textile printing and dyeing industry has led to great concern from all walks of life in the context of the country's in-depth promotion of energy conservation and consumption reduction. The comprehensive development of a low-carbon economy is the fundamental guarantee for China to solve the problem of climate warming and complete the sustainable development of economic development. The traditional textile printing and dyeing industry should also change its development mode to meet the standards of low-carbon economy. Here, the connotation of low-carbon economy and the significance of promoting the low-carbon economic reform of the textile printing and dyeing industry are described, and the current situation and development trend of the low-carbon economy of China's textile printing and dyeing industry is deeply analyzed. Taking the basic theory of garment trade and low-carbon economy as the carrier, the application of low-carbon development mode in China's textile and garment export business process is expounded. According to the fundamental goal of sustainable development of low-carbon economy and related objectives, the adverse impact on the domestic textile and apparel export business process was discussed and eliminated from three aspects: improve the relevant legal system, enhance the development of new energy, and enhance the importance of enterprises in the relevant whole industry chain.

## 1. Overview

Affected by global warming, the Chinese government attaches great importance to the rapid development of the low-carbon economy and regards it as a key step for China to achieve sustainable economic development [1]. At this stage, many enterprises in China still adopt the development model of high-energy consumption and obtain overall economic benefits at the cost of destroying the ecological environment. The literature analysis method is selected for this body activity, which is committed to making the energy consumption mode of factory production more integrated into the requirements of the times, integrating into the reform of the system in our country, accelerating the pace of social reform, and ensuring the main reason for energy conservation and consumption reduction in China. The achievement of this task and overall goal will ultimately ensure the steady development of the physical and mental health of the low-carbon economy in our country. The agricultural emission reduction method is shown in Figure 1 below.

The concept of a low-carbon economy is based on the concept of sustainable development of China's social and economic development. According to a series of countermeasures such as the reform and innovation of industrial production river demonstration points, the application of new energy technologies, and the independent innovation of technologies, fossil energy consumption, carbon emissions, and energy consumption levels can be reduced. This is the overall goal of coordinated development of economic and social development and natural ecological environment [2]. Therefore, from this perspective, the low-carbon economy is not only a new modern economic model but also a strategy to alleviate energy problems and global warming. With the rapid development of the Internet, artificial intelligence, and other technologies, the connotation of low-carbon economy will be further optimized and expanded in economic development and development, covering all aspects of production and manufacturing, commodity circulation, trading, etc.; according to policy innovation, technological reform, and system improvement, the development into a sufficient emphasis on the market economy, to achieve the economy necessary for economic and social development, the key to China's low-carbon economy covers the following aspects [3]. (1) The market model of high energy and low yield in the traditional production industry has been criticized. (2) The low-carbon economy is conducive to the implementation of the clean-up development trend model. The traditional production industry takes fossil raw materials as the basic power energy and a low-carbon economic model with strong carbon emissions, not only to control the consumption of fossil energy but also to develop clean energy technologies and products, actively apply and promote, and balance the relationship between energy consumption and environmental protection. (3) The low-carbon economic model not only needs to use the government to respond to the current policies but also the company needs to improve awareness and increase investment in technical research, in order to obtain the application of the public and change the past high-carbon steel living habits and consumption concepts, so that the low-carbon environmental protection model penetrates into the daily life of the public [4]. In the context of low-carbon emission reduction, the relationship between resources, environment, and economy is shown in Figure 2 below.

## 2. China's Low-Carbon Economy

### 2.1. Development of China's Low-Carbon Economy

In China's government departments, we feel that the green and low-carbon economy is the main step to promote the sustainable development of economic development. As a developing country, China's carbon dioxide emissions are second only to those of the United States, ranking second in the world [5]. In China, due to the lack of related technologies, managers usually choose high-energy consumption methods as the company's development methods from the perspective of funds and network resources. This phenomenon has greatly increased the carbon emissions of Chinese companies. China's ecological environment has long led to nonnegligible destruction. This is also a relatively serious contradiction with the scientific outlook on development that our country has always adhered to. From 28 November to 9 December 2011, the 17th Assembly of States Parties took place in Durban, South Africa. The meeting decided to run the “Emerald Green Climate Equity Fund.” With the development of global climate change negotiations and regular and close cooperation between international economic organizations, China, as a responsible development trend country, should once again assess the carbon emissions of domestic companies and use scientific and technological innovation and industrial structure upgrading to achieve sustainable development of enterprises, reduce carbon emissions, and contribute to the infrastructure of the “global village.” The internal relationship of building a new eco-economic system is shown in Figure 3 below.

China's export commodities have the characteristics of “production and processing” and “low added value” and cannot be linked to the growth rate of import and export trade. The implementation of a low-carbon economy can solve this dilemma and deal with the import and export trade and export problems of enterprises themselves. In the process of energy consumption and ecological environmental protection, China's import and export trade has developed rapidly [6]. The number of commercial disputes arising from environmental pollution problems is increasing. In order to achieve a single ecological and environmental protection purpose, many countries have adopted relevant countermeasures to restrict imports. Relevant trade barriers are more seriously constraining the socioeconomic development of countries in the development trend. Therefore, the development trend of low-carbon economy and the solution of trade barriers are important for Chinese textile trade export companies to gain commercial advantages.

The textile industry is relatively highly dependent on the value of the relevant customers. In China, the textile and garment industry is a labor-intensive field. The industrial model of the “capitalist state factory” [7] is as follows. Through surveys and studies, overseas experts and scholars have shown that China has become one of the important victims of global “economic globalization.” According to the data survey report, in January 2010, under the premise of the smooth recovery of China's textile trade export business process, it was also damaged by the countermeasures related to international economic globalization. In addition, with the trend of economic development globalization and the development of product social division of labor, the improvement of related profits in China's textile industry has shown a weak trend. Experts said that China's textile industry should accelerate industrial transformation and upgrading, promote the transformation and renewal of industrial structure, transform from traditional extensive economic development to green and environmentally friendly low-carbon economic mode, further improve competitive advantages, and enhance trade barriers. The construction of low-carbon ecological cities under the leadership of the government is shown in Figure 4 below.

### 2.2. The Importance of the Textile Printing and Dyeing Industry to Achieve Low-Carbon Economic Development

Due to the aggravation of global warming, the core concept of green economic development must be deeply implemented in the strategic deployment of sustainable development of enterprises [8]. The concept of a green and low-carbon economy includes not only the completion of low environmental standards but also the creation of a low-pollution manipulation management system.

#### 2.2.1. Reduce Production Costs and Improve the Economic Benefits of Enterprises

Energy conservation and emission reduction is an effective way to reduce costs and economic benefits. With the help of cutting-edge technology and equipment, we will integrate technical strength and management capabilities to promote energy conservation and emission reduction and resource utilization and obtain more rights and interests.

#### 2.2.2. Improve the Core Competitiveness of Enterprises in the Market

According to the energy conservation and emission reduction work of the textile industry, some old equipment has been further upgraded and transformed to a new production level. At the same time, the development strategy of energy conservation and emission reduction has been completed, and the overall competitiveness of the textile industry has been obtained in all aspects [9]. At the same time, it is necessary to keep pace with the times to print and dye goods, improve the dyeing and finishing process of textiles using new chemical fibers and new technologies, and improve the postprocessing process such as embroidery patterns, hot stamping, mold making, calenders, bacteriostatic, ultraviolet shielding, coolness, and other multipurpose processes. Implement the fine management of enterprises to cultivate management methods, product added value and market share, enterprise competitive advantages, and competitiveness.

## 3. Low-Carbon Economic Environment for Textile Printing and Dyeing Industry

### 3.1. The Current Situation of Textile Printing and Dyeing Industry in Low-Carbon Economic Environment

The development trend of low-carbon economy and the completion of the modernization and development of “green life and production process” are the goals that all manufacturing enterprises in China need to strive for, and the textile industry is no exception. At this stage, China's textile industry has not been comprehensively rectified. Some small and medium-sized enterprises still use high-energy production and processing technology, but the production volume is low, which is inconsistent with excessive energy consumption, which will cause a major waste of human resources. This objectivity reflects that the slogan of “low-carbon economy” has long been spoken, but it has not really been implemented by printing and dyeing companies [10]. Therefore, China's textile industry has only achieved partial results, and there are a series of problems in the development trend of low-carbon economy. China's long-term low-carbon development transformation goals and paths are shown in Figure 5 below.

#### 3.1.1. Enterprises Have Insufficient Awareness of Low-Carbon Environmental Protection

At this stage, the concept of green environmental protection of enterprises is not enough, and green life is still on the surface. In the raw material supply, manufacturing, marketing, and other aspects, enterprises still use traditional management mechanisms and do not really integrate the core concepts of a low-carbon economy [11]. Therefore, in the field of foreign printing and dyeing, the relevant indicators of the low-carbon economy lack unified standards, and the rational layout of the textile industry is not scientific. In the production system, because of the lack of specific carbon emission indicators and incomplete information, some enterprises refuse to introduce environmentally friendly and low-carbon technology equipment from the first line in order to improve efficiency. The shortage of professional talent pools in the internal structure has constrained the rapid development of the low-carbon economy of enterprises.

#### 3.1.2. Unreasonable Industrial Structure

Since China's reform and opening up, the development concept of giving priority to coastal areas and inland development has won the hearts of the people. Coastal cities are stimulated by the export of foreign trade assets, the economic system is gradually improved, and the range of integrated resources exceeds that of inland areas. Under the premise of promoting regional economic development, it has also caused serious air pollution [12]. Therefore, in response to the key issues at this stage, it is necessary to accelerate the transformation of enterprises, complete the migration of the textile industry in coastal areas to the inland, reduce the development differences in the central and western regions, and promote the transformation and improvement of enterprises. From the perspective of the development of China's central and western regions, there are more natural gas and electricity energy that can be developed in this region, but the development of high-tech and informatization is relatively backward, and the indoor space for development is relatively large. How to make use of the advantages of the central and western regions, develop new energy dominated by photovoltaic and wind power, and improve the rational layout of machinery and equipment of textile printing and dyeing factories are the key development direction, mainly because it can greatly improve product quality and reduce resource consumption. China's national actions in the midst of a low-carbon transition are shown in Figure 6 below.

#### 3.1.3. High-Energy Consumption

China has taken the initiative to remediate its own companies, but it consumes more electricity and energy than more developed countries. In China's textile industry, there are many problems such as long industrial chain, long production and manufacturing time, high-energy consumption, and long-term wastewater treatment, which seriously endanger the energy consumption of industrial production in China. China's low-carbon environmental protection development has encountered new challenges, and the development of green and low-carbon economy in the textile industry is more difficult [13] At this stage, many countries have implemented “carbon tariffs.” In the future, in China, we will conform to the trend of the times and use corresponding countermeasures to manipulate the utilization of coal energy and further restrain the development of the textile industry.

#### 3.1.4. Oversupply in the Textile Industry

Chinese mouths are very large, but there is always an unbalanced system between the manufacturing system and the trading system of the textile industry, that is, oversupply. In order to obtain relevant profits, it is necessary to export a lot of textile products [14] Part of the textiles is the domestic resources produced and manufactured, many of which consume limited resources. The state has introduced the current policy of accelerating the replacement of some backward production capacity enterprises and technologies, but the corresponding problems such as outdated machinery and equipment, low production and manufacturing efficiency, and insufficient staffing have not been dealt with in essence, which limits printing and dyeing: the development of the industry and the pace of China's development trend towards a “green and low-carbon economy”.

### 3.2. Development Trend of Textile Printing and Dyeing Industry under Low-Carbon Economy

#### 3.2.1. Enhance Enterprises' Awareness of Low-Carbon Environmental Protection

1. Executives of textile printing and dyeing enterprises should fully understand the necessity of developing a low-carbon economy. In order to achieve the goal of low-carbon economy, enterprises must draw low-carbon economic concepts from the level of research and development technology, manufacturing, marketing, etc. and follow the low-carbon economic norms promulgated by the national and local governments to promote the development of the entire textile industry in a green and healthy direction. From the perspective of short-term economic benefits, this transformation is a huge project investment, which brings huge financial and human resources pressure to large, medium, and small textile printing and dyeing enterprises [15]. However, with the times, under the concept of low-carbon economy, the energy consumption of enterprises continues to decline, and various costs are also reduced accordingly, coupled with the development and marketing promotion of new low-carbon textile products, which can meet the market's needs for low-carbon textile products. The demand for new carbon products will drive the company's sales and profit growth, laying the foundation for the company's long-term steady development based on the market share of the product
2. The rise of textile printing and dyeing enterprises: in the process of changing to low-carbon and efficient production methods, it is necessary to strengthen the low-carbon economy publicity and planning of the bottom employees and shape their scientific and reasonable low-carbon concepts, so that employees in all positions of the enterprise in the premise of mastering low-carbon production and manufacturing, starting from themselves, in the work and life of the serious implementation of the low-carbon concept are as follows. At the same time, enterprises can also cooperate with industry associations to enhance the publicity of low-carbon knowledge and low-carbon environmental protection quality of employees
3. In order to enhance the low-carbon environmental awareness of textile enterprises, government departments can give certain financial subsidies in policies to reward those enterprises that meet the standards in low-carbon technology research and development and production and enhance their enthusiasm for developing a low-carbon economic model. China's carbon reduction plan is shown in Figure 7 below

#### 3.2.2. Improve Industry Laws and Regulations

At this stage, the relevant laws and regulations of the textile printing and dyeing industry in China's green and low-carbon economy are not perfect, and many enterprises in the industry are deeply trapped in the dilemma of basing on the current policies and norms [16]. Therefore, the relevant departments should create a policy system according to the specific development orientation of the industry, implement the energy-saving and emission-reduction measures of the textile printing and dyeing industry, comprehensively test the low-carbon and environmental protection development of textile products, and encourage the development of textile products to the direction of high efficiency and low consumption [17]. The printing and dyeing industry is relatively developed, and some local governments in Zhejiang have introduced new policies to promote the overall transformation and development of enterprises in the region and develop towards ecology, intelligence, and branding. The government department first set up a new platform for cooperation and innovation. The changes in the printing and dyeing industry “take the pulse”, provide solutions, cultivate a large number of well-known and excellent enterprises at home and abroad, and strive to create a modern industrial cluster of “emerald green high-grade and leading technology.”

#### 3.2.3. Trends in Change

The textile industry has played an extremely important social role in China's green environmental protection industry and shoulders a huge corporate social responsibility. Under such circumstances, in China's large, medium, and small textile printing and dyeing companies, it must use the relevant national policies and the use of national project investment, to achieve their own technical equipment requirements and product quality. Some small and medium-sized textile enterprises can learn from large- and medium-sized textile enterprises about textile printing and dyeing technology and cooperate with well-known enterprises to complete intelligent production and manufacturing. According to China's “Belt and Road” initiative, it can shape well-known brands with Chinese characteristics and produce distinctive well-known brands such as Chinese qipao skirts, Zhongshan costumes, and ancient clothing and grow the brand. In this regard, we have actively promoted the application of energy-saving and consumption-reducing methods in the chemical fiber printing and dyeing industry, created a green economic management system, improved the production technology of the factory, and overcome many difficulties faced in the field of chemical fiber printing and dyeing.

#### 3.2.4. Attach Importance to Talent Development

To implement the concept of low-carbon economy into the production and marketing of printing and dyeing enterprises, it is necessary to support high-quality talents. High-quality talents are the energy of internal reform and development of enterprises, which means that the image of enterprises opening up to the outside world is the meaning. Under the premise of vigorously investing in new environmental protection equipment and innovative production processes in projects, textile enterprises must control and supervise the literacy of employees in the internal structure, organize employees on time, and build a key cohesion within the enterprise, so that employees can fully use their own value under the concept of low-carbon economy. Companies must also provide employees with a different and innovative environment, so that employees can independently and freely express their ideas and opinions, and show their own level according to their own understanding of the low-carbon economy. On this basis, an incentive mechanism can be adopted to motivate employees to actively carry out the basic construction of the enterprise, improve the internal structure of the enterprise, and attract talents with generous remuneration. In addition, enterprises should also dig deep into the development potential of employees and give employees green environmental protection professional skills on time, so that employees can grasp the latest low-carbon economy manufacturing concepts and better integrate into their posts.

#### 3.2.5. Increase Support for Low-Carbon Emission Reductions

1. For textile printing and dyeing enterprises, the development trend of low-carbon economy is not only the banner of reform and innovation but also the inherent requirement of industry development. Therefore, government departments should increase support for low-carbon, energy-saving, and consumption-reduction. First of all, the government should guide tester printing and dyeing enterprises in a key and correct manner, stimulate the research and development of low-carbon technologies and low-carbon products, encourage active funds to invest in new technology applications and new product research and development, and implement a series of incentive mechanisms [18]. Second, government departments should give full play to their own advantages, through collaboration with low-carbon technologies in developed countries, introduce the most advanced low-carbon technologies, promote the development trend of China's low-carbon economic mode, and correctly guide China textile printing and dyeing companies to move towards a low-carbon economy. The changes in China's carbon dioxide emissions from 2016 to 2020 are changed in Table 1.

(2) The research and development of low-carbon technologies and products must be applied with a large amount of funds, but in the field of textile printing and dyeing in China, small- and medium-sized enterprises are the core, and the profitability is medium. Therefore, government agencies must take corresponding countermeasures to help enterprises carry out the financing process and reduce financing costs. For example, for the textile industry, which has a better effect on energy conservation and consumption reduction, government departments can provide relatively high belief lines and obtain information appropriately to help enterprises implement low-carbon reform and innovation. In recent years, many regions in China have established emerald green carbon funds, the purpose of which is to promote the flow of market funds to projects such as carbon sinks, afforestation, and forest resource protection in the forest and fruit industry. At the same time, it can also promote the capital construction of low-carbon textile industry securities funds, manipulate the flow of funds, improve the concept of carbon sinks of the masses, and provide financial support for the development trend of low-carbon development in the field of textile printing and dyeing
(3) Government departments can carry out pilot work with symbolic companies with strong overall strength. The textile printing and dyeing mill industry has established low-carbon product verification standards, covering all stages of textile printing and dyeing products from raw material production and manufacturing to market consumption. The specific quantitative analysis of carbon emission standards in the whole process is conducive to improving the operation and management of enterprises in the industry in the production, supply, and marketing stage, achieving the specified energy conservation and emission reduction standards, and controlling air pollution. After the establishment of industry verification standards for low-carbon products, it meets the international high standards for low-carbon products and domestic textile printing and dyeing industry standards, which can promote low-carbon social and economic development. The estimation of China's decarbonization path in 2060 is shown in Table 2 below

#### 3.2.6. Optimize the Energy Structure and Improve Energy Utilization

Because coal energy is rich and colorful in China, it is impossible to change the current situation of energy consumption in most industries in China in a short period of time, and it is impossible to improve the energy consumption structure of China's textile industry.

First, it is necessary to control the total consumption of high-carbon fossil fuels (usually coal carbon) and develop clean coal technologies. Therefore, we should attach great importance to scientific research and development and coal-based fossil energy efficiency and make the application of fossil energy more clean and efficient, so as to achieve the effect of energy saving and consumption reduction [19]. Secondly, because fossil energy is nonrenewable, in response to the reduction of nonrenewable resources, the research and development of renewable resources have also become the focus of human attention, which is related to the future survival and development of mankind. Renewable resources such as wind speed, solar power generation, and hydropower projects are mostly found in clean energy, and China's undeveloped renewable resources have great potential. Therefore, it is beneficial to enhance the automation development, design and utilization of clean energy, enhance the relevant industrial equipment of the textile industry, complete the industrialization of clean energy as soon as possible, gradually replace fossil energy, and promote the rapid development of the green and low-carbon economy in the textile industry.

Ultimately, in order to promote the development and utilization of clean energy, it is necessary to accelerate the operation of China's carbon emissions trading market. After the market-oriented operation, the carbon emission quota of textile enterprises will be combined with the energy consumption structure of enterprises and new energy technology to accelerate the energy conservation and consumption reduction of textile enterprises. On the one hand, improve the structure of energy consumption, promote textile enterprises to introduce the technicality of cleaning up fossil energy, control air pollution, promote transformation and development, and reduce costs. On the other hand, reduce the transaction cost of carbon emission allowances, save the quota system according to the sale and purchase, and improve the economic benefits that George brings to the enterprise. This will well stimulate the enthusiasm of textile enterprises to develop a low-carbon economy.

## 4. The Impact of Low-Carbon Economy on China's Textile and Garment Exports and Countermeasures

### 4.1. Low-Carbon Economy Puts Forward Strict Requirements for the Costs Related to China's Textile and Garment Exports

Affected by the low-carbon economic plan, the Chinese government has given low-carbon regulations on the whole process of exporting garment and textile products, that is, to reduce the carbon emissions of such commodities in the production, application, and disposal process in an all-round way, so that the discharge of pollutants can meet relevant national standards. However, in the practice of reducing the carbon emissions of related processing processes, many Chinese companies have found that they lack sufficient low-carbon machinery and equipment. The main reason is that due to the impact of the financial turmoil, the wages of employees, the cost of renting venues, related raw materials, and other factors have increased. The relative cost advantages of new products in China's textile trade have weakened. Responding to the financial crisis has consumed a lot of time and energy of Chinese textile export-related companies. Therefore, if we invest in the project to increase capital to purchase “low-carbon” hardware allocation and reduce related carbon emissions, it will further reduce the cost advantages of China's textile and apparel export business. Therefore, how to maintain the cost advantage has become an urgent problem to be solved in China's textile and garment export companies.

### 4.2. The Low-Carbon Economy Puts Forward Higher Requirements for the Relevant Technologies of China's Textile and Garment Exports

Green and low-carbon economy harms the cost of textile and apparel commodities in China, but more importantly, to achieve technological progress in production. According to the relevant basic theories of development economics, the technological progress of enterprises is often closely related to the stimulation of environmental factors. Without external stimulus, the technology development trend of enterprises is generally gradual. The introduction of external pressure such as market competition can well stimulate the enthusiasm of enterprises in work and innovation and promote the development trend of enterprise technology to complete leapfrog development. In China, the relevant production line equipment of textile and garment production and manufacturing enterprises often needs to be imported from other countries; so, the overall production and manufacturing level and production technology lag behind capitalist countries to a certain extent. The birth of this phenomenon shows that the production technology of textile and garment in China needs to be developed.

### 4.3. Countermeasures to Address the Adverse Effects of a Low-Carbon Economy

#### 4.3.1. Improve the Relevant Legal System

The government's overall planning for national development can provide the necessary for the sustainable development of the low-carbon economy to ensure that China's current relevant laws and regulations on energy conservation and consumption reduction mainly include the Energy Conservation Law and the Renewable Energy Law. However, these existing legal systems are not enough to meet the development provisions of a low-carbon and environmentally friendly society. Therefore, the government should appropriately learn from the successful cases of capitalist countries in solving related problems, further promulgate major policies related to the low-carbon economy, create efficient laws and regulations and policies in many aspects such as enterprise environmental protection, environmental protection and energy conservation, and new energy technology, and closely integrate them. The specific development trend of relevant enterprises in China has given a higher demand for corporate carbon emissions specifications [20]. On the other hand, the government should educate and guide relevant enterprises through macroeconomic policy countermeasures, increase capital investment, and encourage textile export and garment enterprises with economic strength to accelerate the introduction of new technology applications, purchase of new machines and energy-saving technologies. Related enterprises that are not basically competitive should be appropriately replaced. For a regional comparison of national carbon emissions trading prices from 2013 to 2018, see Table 3.

#### 4.3.2. Strengthen the Development and Utilization of New Energy Sources

With the times, measures such as low-carbon energy conservation and emission reduction regulations and carbon tariffs will stimulate the production processes of export enterprises to use cleaner energy-saving and emission-reduction technologies for production and trade. At present, many textile and garment production enterprises in China use traditional network resources such as coal as the only power energy source in the production process, which has led to serious environmental pollution to the environment. Therefore, China will fully implement the utilization of new energy technologies, increase the capital investment of relevant government departments, actively develop the development trend of solar power, wind power, solar power, tidal power and other clean-up environmental protection energy, and correctly guide China's textile and garment production enterprises to use carbon emissions from traditional network resources such as coal and crude oil. On the basis of understanding the low-carbon economy, China's textile and garment production enterprises should strengthen scientific research on machinery, equipment, technology, and processes in textile and garment production. The company can improve the production process by introducing new technologies and adjusting the industrial structure. According to the data survey report, most of the clothing imported and exported in Europe and the United States is the commodity entrusted by investors to process materials, and more than 80% of the profits are still obtained by buyers in Europe and the United States. Coupled with the impact of the low-carbon fortress, the profits of China's textile and garment companies in this process will be reduced. Therefore, the company can only give full play to its own advantages, introduce new technologies, develop new power energy, formulate new standards, develop new commodities, and build competitive advantages in order to gain a firm foothold in global competition.

#### 4.3.3. Improve the Position of Enterprises in the Relevant Industrial Chain

Domestic textile companies are mainly processing companies, which are at the low end of the industrial chain and obtain relatively low production costs in the production and installation of commodities. During processing, commodities generally have greater air pollution.

What is more serious is that the carbon emissions are larger than other links, and the benefits are smaller than other links. In contrast, high-end products such as design solutions and marketing have basically no carbon emissions and are more profitable. Therefore, in China's textile export and garment-related enterprises to accelerate the transformation of industrial structure and heightened footsteps and actively carry out the design of products, marketing, and other aspects of the industrial chain-related work, from the low-end link of the industrial chain to the high-end link, international government departments between the negotiation and consultation must win the company's development dominance, to complete the green barriers.

## 5. Summary

In the process of China's textile export and garment, according to the sound of the corresponding legal system, they must encourage outstanding enterprises to develop technology, according to the comprehensive utilization of new energy technology and new technologies, reasonably reduce the carbon emissions of Chinese enterprises, get rid of green barriers, enable enterprises to further solve the dependence on alternative fuels, reduce the pressure of increasing costs of enterprises affected by the financial crisis, escort enterprises to exert their own advantages, create competitive advantages, and provide technical support for enterprises to cope with more fierce global competition. The rapid development of the low-carbon economy has added great pressure to the survival of printing and dyeing enterprises in China, which is a key opportunity for development and reform. Textile enterprises want to achieve long-term development in the market economic system and must follow the trend, in line with the development trend of China's green development infrastructure, in all aspects of the internal structure of the enterprise and management mechanism to seriously implement the concept of low-carbon economy, with the help of research and development technology to create their own brand, in order to occupy a place in the market.

Low-carbon environmental protection and ecological environmental protection have become the trend of social development and development. Actively implementing the current policy of low-carbon environmental protection can enable textile engineering enterprises to keep up with the pace of the times and actively act. Textile enterprises should improve technology and production processes, take the initiative to develop and design new sustainable energy and raw materials, and promote independent innovation while generating the core competitiveness of textile floor tile project enterprises. Under the concept of green environmental protection, textile engineering enterprises can not only reduce energy consumption, emissions, and environmental pollution but also enable textile engineering enterprises to effectively save costs in the development process and at the same time pass on the concept of green environmental protection to the masses.

## Figures and Tables

**Figure 1:** Green emission reduction methods.

**Figure 2:** Relationship between resources, environment, and economy under the background of low-carbon emission reduction.

**Figure 3:** Internal relations of building a new ecological and economic system.

**Figure 4:** Construction of low-carbon ecocities under the leadership of the government.

**Figure 5:** China's long-term low-carbon development transformation goals and paths.

**Figure 6:** National actions for China's low-carbon transition.

**Figure 7:** Timeline of carbon reduction in China.

**Table 1:** CO_2_ emissions in China from 2016 to 2020.

Year	2016	2017	2018	2019	2020
China's carbon dioxide emissions (100 million tons)	92.74	94.63	96.69	98.06	98.94

**Table 2:** Estimation of China's decarbonization path in 2060.

Year	2020	2030	2040	2050	2060
Carbon removal rate (gigatons)	11	11.5 _ _	8	5	2

**Table 3:** Regional comparison of national carbon emissions trading prices from 2013 to 2018.

City	Beijing	Shanghai	Shenzhen	Guangdong	Tianjin
Transaction Price (RMB)	8.87	2.44	20.00	8.97	11.18

## Data Availability

The labeled data set used to support the findings of this study is available from the corresponding author upon request.

## References

[1] Feng D. (2022). Analysis on the status quo and development of textile printing and dyeing industry under low-carbon economic environment. *Textile Report*.

[2] Fahmy H. M. (2021). Overview of China's textile and clothing foreign trade in the first half of 2021. *China Textile (English version)*.

[3] Guangyi A. (2021). Analysis of the impact of low-carbon economy on china's textile and apparel exports. *Textile Industry and Technology*.

[4] Badri (2018). Better development ahead for China's textile export in 2018. *China Textile (English version)*.

[5] Qing M. (2021). Current situation and development trend of textile printing and dyeing industry under low-carbon economy. *National Circulation Economy*.

[6] Saheed H. (2018). Prospects for the textile and clothing industry in China. *Textile Outlook International: Business and Market Analysis for the Textile & Apparel Industries*.

[7] Meixin S. (2019). The impact of low-carbon barriers on my country's textile and apparel exports and countermeasures. *Reform and Opening*.

[8] Saheed H. (2020). Prospects for the textile and clothing industry in South Korea. *Textile Outlook International: Business and Market Analysis for the Textile & Apparel Industries*.

[9] Liping W. (2021). Countermeasures for the development of China's textile and garment foreign trade enterprises under the low-carbon economy. *Chemical Fiber and Textile Technology*.

[10] Saheed H. (2019). Prospects for the textile and clothing industry in China. *Textile Outlook International: Business and Market Analysis for the Textile & Apparel Industries*.

[11] Lijie L., Cuncun T. (2020). On the status quo and development trend of low carbon economy in textile printing and dyeing industry. *Shandong Textile Economy*.

[12] Kanat S. (2019). Analysis of the competitiveness of the Turkish textile and clothing sector in the European Union market. *Fibres & Textiles in Eastern Europe*.

[13] Tao Z. (2022). *Status quo and development trend of textile printing and dyeing industry under low-carbon economy*.

[14] Ding Y., Yu H. (2022). Low carbon economy assessment in china using the super-SBM model. *Discrete Dynamics in Nature and Society*.

[15] Lal K., Mohnen P. (2018). Innovation Policies and International Trade Rules: The Textile and Clothing Industry in Developing Countries. *The European Journal of Development Research*.

[16] Meixin S. (2019). *Status quo and development trend of low carbon economy in textile printing and dyeing industry*.

[17] Lili N. (2020). China's textile and apparel industry is advancing under pressure in 2020. *China Textile (English)*.

[18] Siyi W. (2018). Analysis on the development path of low-carbon textile economy. *Textile Report*.

[19] Adeel S., Rizwan E. M., Urooj N., Musawir S. A. (2022). Forecasting practices in textile and apparel export industry. *International Journal of Circular Economy and Waste Management (IJCEWM)*.

[20] Laua Y.-Y., Chanc M.-H., Nguyen H.-O. (2017). China's textile and clothing case and OBOR implications. *Journal of International Logistics and Trade*.

